# Optimal Design of International Trade Logistics Based on Internet of Things Technology

This article has been retracted.

**DOI:** 10.1155/2022/8781095

**Published:** 2022-04-07

**Authors:** Yue Wang

**Affiliations:** College of Economics and Management, Guizhou Institute of Technology, Guiyang 550003, Guizhou, China

## Abstract

With the global industrial integration, trade exchanges between countries are becoming more and more frequent and the competition for related international trade logistics is becoming more and more intense. This paper aims to study the optimization design of international trade logistics based on Internet of Things technology. For this reason, this paper proposes an RFID method, through which it is possible to master a journey in the actual international trade logistics process. And it optimizes and improves its related paths, shortens the time delayed on the road, and achieves the purpose of mentioning the carrying capacity. And for the actual use effect, the relevant experiments and analysis parts are designed to simulate it. The experimental results of this paper show that the improved and optimized international trade logistics shortens the carrying time by 28.6% and increases the carrying capacity by 34.2%, which greatly promotes the development of the relevant international trade logistics industry.

## 1. Introduction

The continuous development of the contemporary world economy toward integration has greatly promoted the development of international trade and international shipping, and logistics has played an increasingly powerful role in the development of the regional economy. After realizing the importance of logistics, all parts of the world are actively developing the logistics economy, and the competition among logistics is becoming more and more fierce, which makes the development of logistics more inclined to the specialization of functions, large-scale scale, modernization of technology, and scientific management. These changes make the competitive environment among logistics more cruel, but at the same time promote the rapid development of logistics in a better and more efficient direction.

Through the analysis of the construction of the existing international trade logistics platform, the development of international trade logistics has accelerated the operation of enterprise logistics, and it is also beneficial to the development of international trade. On the one hand, it can improve the loading and unloading processes, reduce the production cost, and improve the economic benefits of international trade, which is beneficial to the long-term development of international trade; on the other hand, it enhances the expansion function of international trade, extends the basic function of international trade, and provides a new economic growth point for the development of international trade, thereby reducing the operational risk of international trade. From the perspective of international competition, the development of international trade logistics can help to establish an international trade logistics center and improve the comprehensive benefits of international trade logistics.

The innovation of this paper lies in the use of the key technology of the Internet of Things, that is, RFID radio frequency technology. And the technology is optimized so that the improved RFID technology can be better applied to the research topic of this paper. And the relevant national trade logistics is also analyzed and researched, and its memory is optimized and improved to a certain extent.

## 2. Related Work

With the development of economy and the expansion of globalization and internationalization, international trade logistics does not meet the basic functions of simple loading and unloading, warehousing, and so on. How to adapt international trade logistics to the requirements of modern development, how to promote the sustainable development of economy and trade, and how to promote the regional development of surrounding areas have become one of the urgent problems to be solved. Lai M proposes a vehicle initial path optimization model considering uncertainty, considering vehicle capacity, customer time window, maximum travel distance, and road capacity [1]. The model proposed by Zhang et al. is formulated as a two-layer formula in which the upper layer determines the optimal choice of logistics infrastructure investment and green transportation mode subsidies to maximize the benefit-cost ratio of the entire logistics system [2]. Based on the relationship between suppliers, transit warehouses, and sellers in the collaborative logistics network, Xu et al. established a two-level programming model with random constraints considering the uncertainty of time. He proposed a genetic simulated annealing mixed intelligence algorithm to solve it. Numerical examples show that the method has strong robustness and convergence, and it can realize the rationalization and optimization of resource allocation in collaborative logistics network [3]. Aiming at the common distribution methods of urban logistics in the e-commerce environment, Yang considers the dynamic uncertainty of the urban road network based on the optimization of the distribution path [4]. Liu et al. proposed a stochastic model of postdisaster relief logistics to guide the tactical design of mobilizing relief material levels, planning initial helicopter deployments, and creating transport. He introduced a robust optimization method to deal with these uncertainties and derived a robust counterpart of the proposed stochastic model [5]. Rajasekar et al. reconsidered the problem of conflicting optimization goals, focusing on low inventory levels and short throughput times. It generates conversions of some performance metrics (such as delivery time and latency) to penalties. When manufacturing is the main economic activity of an industry, changes in production patterns pose challenges to the logistics system, forcing manufacturers to optimize the logistics system [6]. Dossou and Vermersch defined a study based on a cocreation approach that integrates all stakeholders (local authorities, companies, and citizens) to develop alternative solutions for road transport. It is used for the architecture and development of decision aids for simulating and optimizing alternative solutions to road traffic [7]. Malladi and Sowlatti proposed that biomass logistics was reviewed in a previous study aimed at classifying logistics operations, but the inherent issues and complexities and how they were incorporated into mathematical models were not discussed in detail. Their aim is to review the important features of biomass logistics operations, discuss how to incorporate them into mathematical optimization models, and explain new trends in biomass logistics optimization [8]. The above-mentioned literature is very good for the relevant logistics optimization ideas, and the relevant technical explanations are all in place. The proposed model is also studied in detail. However, the Internet of Things technology is not used in a certain combination, and the introduction of the relevant experimental process is not detailed enough.

## 3. International Trade Logistics Optimization Method

### 3.1. IoT Technology

#### 3.1.1. Concept of Internet of Things

At present, there is still no authoritative definition of the Internet of Things. From the technical field, the Internet of Things refers to the integration of various technologies (sensors, wireless sensors, smart embedded, Internet, RFID, smart processing, nano, etc.), and through the Internet of Things, the interconnection of all things can be realized. It has the characteristics of precise control, reliable transmission, and comprehensive processing intelligence and perception.  Figure 1 shows a typical IoT structure diagram [9].

#### 3.1.2. IoT Architecture

The Internet of Things technology includes computer and Internet technology. It identifies and manages physical objects through modern information technology and uses wireless communication technology to achieve information exchange [10]. The Internet of Things has obvious advantages, the most notable feature of which is that it greatly reduces production costs while improving economic benefits. The Internet of Things is usually divided into five parts, namely, readers, electronic tags, Internet of Things name resolution servers, Internet of Things middleware, and Internet of Things information publishing services.

At present, the Internet of Things is at the forefront of technology, the technology is strict and complex, and the technology is not mature enough [11]. From the analysis of the current application requirements of the Internet of Things, the academic community generally divides the Internet of Things into three levels (1. perception layer; 2. network layer; and 3. application layer) as shown in Figure 2.

Perceptual recognition technology is the core technology of the Internet of Things [12]. The perception layer is mainly composed of various sensors and their gateways, which are mainly used to collect data. Its specific data indicators include various types of digital data, video data, audio, and identification [13]. The key technologies of IoT data collection include sensor technology, RFID technology, multimedia information collection technology, two-dimensional code technology, and real-time positioning technology. Taking people as an example, the nerve endings of human sensory eyes, ears, throat, nose, and skin are equivalent to the perception layer mentioned above. In the Internet of Things, identifying objects and collecting information sources is the core function of the perception layer [14].

The three compartments in the Internet of Things are independent of each other, but there is a close connection between the three compartments. In the introduction to the network layer, people are also taken as an example. The network layer can be compared to the human nerve center, which is responsible for transmitting and processing the digital information taken by the perception layer. The technical functions on each compartment complement each other and play different roles according to different environments to adapt to different application environments, thus forming a complete coping strategy for the compartment technology [15]. The security technology, identification and analysis, service quality management, and network management in the public technology are related to the above three layers of the IoT architecture to a certain extent, but they do not belong to a specific layer in the IoT technology.

#### 3.1.3. Perception Layer Functions and Technologies

In view of the large amount of information obtained through perception functions, there is a large demand for geographic and spatial scope. The devices in the perception layer also need to form a self-organizing multinode network in a cooperative manner, and transmit data through the self-organizing network technology [16]. To realize the sensing function, the sensor network firstly touches and senses the sensed object in all directions through different sensors, and then comprehensively identifies and analyzes the acquired sensing data.

#### 3.1.4. Key Technologies of the Perception Layer

RFID tags contain electronically stored information, so they can be identified within a few meters. Some tags do not need energy themselves and obtain energy from electromagnetic fields during identification; some tags themselves have power or energy, which can actively generate radio waves, the so-called electromagnetic fields tuned to radio frequencies. RFID technology has been used in most industries today [17]. Car manufacturers can know the progress of the car on the production line based on the label on the car, and the warehouse can also know the information of the goods in real time. In addition, radio frequency tags can also be applied to animals to facilitate the positive identification of animals. The radio frequency transponder installed on the car can be used to collect parking fees and also can be used to collect road tolls. Of course, this technology has the possibility of obtaining personal information without the consent of the individual, and this technology will infringe on the privacy of others to a certain extent [18].

The RFID application system is mainly used to control, detect, and track objects. The principle of RFID is not complicated, its application system principle is actually very simple, the composition is also simple, and it is composed of two basic devices. The system consists of an interrogator, the so-called reader, and many transponders [19]. Its basic composition is shown in Figure 3.

Signal receivers also exist in RFID systems, which are often referred to as readers. The sophistication of readers varies widely based on the types of tags supported and the capabilities they perform. Its main function is to provide a data transmission method.

Receiving the radio frequency signal sent by the reader, the tag relies on the energy obtained by the induced current to send out the product information stored in the chip, or the tag can actively send a signal of a specific frequency. After reading and decoding the information, the reader sends the data and information to the central information system for further processing [20].

The signal transmitter exists in the RFID system, and its existing forms are also different according to the requirements of the application, and the label is its typical form. The tags include antennas, coils, memory, and low-power integrated circuits for control systems. The role of the label is like a barcode, and its role is to store information [21]. However, compared with barcodes, it has the characteristics of actively transmitting information [22]. The salient feature of RFID tags different from barcodes is that they do not need to be placed in the line of sight of the identifier, and RFID tags can also be embedded in the tracked object.

### 3.2. Power Transmission of the RFID Real-Time Positioning System

In order to analyze the link characteristics and system indicators of the system, it is necessary to quantitatively analyze the power transmission mechanism of the RFID real-time positioning system. This includes the analysis of the path loss characteristics of the channel and the reflection characteristics of the tags. It first analyzes the path loss characteristics of the system.

The RFID system is a short-range wireless communication system, and the path loss of the system can be analyzed using the free space propagation model [23]. Assuming that the transmitting power of the reader is, it is transmitted outward through the antenna with a gain of. It can be seen from the formula that the relationship between path loss and distance is as follows:

(1) $$\begin{array}{c} P_{\text{channel}}|{}_{dB}=20\;\log\left(\frac{\lambda }{4\pi d}\right). \end{array}$$

It can be known from the above formula that the maximum linear dimension D of the cross section of the transmitting antenna is related to the wavelength. Fraunhofer distance is defined as

(2) $$\begin{array}{c} d_{f}=\frac{2D^{2}}{\lambda }. \end{array}$$

Let *h*_1_ be the height of the reader, *h*_2_ the height of the tag, and *d* the horizontal distance between the reader and the tag. *E*_tag_ is the electric field strength received by the tag, and its expression is as follows:

(3) $$\begin{array}{c} \left|E_{tag}\right|=2\cdot \frac{\sqrt{30\cdot \text{EIRP}}}{d}\cdot \;\sin\left(\frac{2\pi h_{1}h_{2}}{\lambda d}\right). \end{array}$$

Assuming that the EIRP is 4 W, the height of the reader and the tag are both 1 m, and the signal power received by the tag can be expressed as

(4) $$\begin{array}{c} P_{tag}=\frac{{\left|E_{tag}\right|}^{2}\lambda^{2}}{480\pi^{2}},\\ P_{tag}=\sin^{2}\left(\frac{2\pi }{\lambda d}\right)\cdot {\left(\frac{\lambda }{d\pi }\right)}^{2}. \end{array}$$

When the effective transmit power of the reader is 4 W, the received signal power obtained according to the free space attenuation model is as follows:

(5) $$\begin{array}{c} P_{\text{tag}}^{\prime }=4\cdot {\left(\frac{\lambda }{4\pi d}\right)}^{2},\\ P_{\text{tag}}^{\prime }=\frac{1}{4}{\left(\frac{\lambda }{\pi d}\right)}^{2}. \end{array}$$

As shown in Figure 4, the relationship between the received signal power of the tag and the distance obtained under the two models is given.

According to the working principle of the UHF RFID system, the energy received by the tag is roughly divided into two parts. One part is received by the tag antenna, enters the tag chip, and is rectified for the tag to work, and the other part is backscattered by the tag antenna [24]. To quantify the energy distribution between received and reflected, the tag antenna and tag chip can be modeled as shown in Figure 5.

*v*_*s*_ and *I*_*s*_ in the figure represent the peak voltage and peak current that can be induced by the tag antenna when it is not loaded; *z*_*A*_ represents the impedance of the tag antenna, *z*_*L*_ represents the impedance of the tag chip, and there are as follows:

(6) $$\begin{array}{c} Z_{A}=R_{A}+jX_{A},\\ Z_{L}=R_{L}+jX_{L}. \end{array}$$

Then, the reflection coefficient of the label is defined as

(7) $$\begin{array}{c} \Gamma =\frac{Z_{L}-Z_{A}^{*}}{Z_{L}+Z_{A}}. \end{array}$$

Then, the power that can be obtained by the tag is as follows:

(8) RRF,in=12ReVS∗·IS.

Available power is as follows:

(9) $$\begin{array}{c} R_{\text{RF,in}}=P_{\text{avail}}\left(1-{\left|\Gamma \right|}^{2}\right), \end{array}$$

where

(10) $$\begin{array}{c} P_{\text{avail}}=\frac{V_{S}^{2}}{8R_{A}}. \end{array}$$

The load impedance of the tag during normal operation switches between two impedances is as follows:

(11) $$\begin{array}{c} Z_{1}=R_{1}+jX_{1},\\ Z_{2}=R_{2}+jX_{2}. \end{array}$$

The reflection coefficient and the power received by the tag also vary between the two states with

(12) $$\begin{array}{c} R_{\text{RF,in,}1,2}=P_{\text{avail}}\left(1-{\left|\Gamma_{1,2}\right|}^{2}\right). \end{array}$$

Assuming that the probabilities of the two states appearing are *P*1 and *P*2, respectively, the average available power received by the tag is as follows:

(13) $$\begin{array}{c} P_{\text{RF,in,ave}}=p_{1}P_{\text{RF,in,}1}+p_{2}P_{RF,in,2}. \end{array}$$

In order to calculate the power reflected back by the tag antenna, the resistance of the antenna can be divided into two parts: radiation resistance *R*_*ra*  *d*_ and lossy resistance *R*_*loss*_, namely,

(14) $$\begin{array}{c} Z_{A}=R_{A}+jX_{A},\\ Z_{A}=R_{\text{loss}}+R_{\text{rad}}+jX_{A}. \end{array}$$

The current flowing through the antenna as the tag changes between the two states is as follows:

(15) $$\begin{array}{c} i_{1,2}=\frac{V_{S}}{Z_{A}+Z_{1,2}}. \end{array}$$

Suppose the two states are equally likely to occur, both are as follows:

(16) $$\begin{array}{c} p_{1}=p_{2}=0.5. \end{array}$$

Then, the signal power reflected by the tag is as follows:

(17) $$\begin{array}{c} P_{bs}=\frac{P_{\text{avail}}}{4L_{A}}{\left|\Gamma_{1}-\Gamma_{2}\right|}^{2}. \end{array}$$

### 3.3. International Trade and International Logistics

With the development of international trade, international logistics has been continuously improved. As a bridge of economic exchanges between countries, international logistics and international trade together constitute two indispensable aspects of international economic development [25].

Generally speaking, international logistics mainly face three barriers (Market and Competition, Financial Barriers, and Distribution Channels), as shown in Figure 6. The development of international logistics must balance the relationship between the actual cost of overcoming these barriers and the potential benefits of international trade, in order to obtain actual benefits through successful international operations.

Market and competitive barriers: market and competition barriers in international logistics mainly refer to market entry restrictions, information symmetry, pricing, and competitive environment [26].

First, market entry restrictions often create market entry barriers for imported goods through legislation or judicial practice.

Second, information symmetry is another barrier to international logistics. In addition to information asymmetry about market size, population, and competition conditions, the information used to clarify import operations and related documents is often not coordinated [27].

## 4. RFID Experiment Based on IoT

### 4.1. Distribution and Transportation Experiment

In the international trade logistics, the logistics distribution center plays a linking role. Its upstream is international processing enterprises, and its downstream is major users. The international processing enterprise sends the processed products to the warehouse of the distribution center, and the distribution center completes the distribution of the processed products through transportation vehicles according to the requirements of customers. Because of the particularity of international trade logistics, enterprises are required to maintain a reasonable placement of finished products in a series of processes (warehousing and warehousing, loading and unloading, and distribution and transportation). The data collected during the distribution and transportation process and the corresponding equipment are shown in Table 1:

### 4.2. Example Application Experiment

The calculation of genetic algorithm can be performed by the computer to verify its effectiveness in the optimization of cold chain logistics distribution path. With the help of Matlab 2011a, by writing the corresponding computer program of the model, the genetic algorithm is used to calculate the model, and the optimal solution of the problem is obtained. Taking city A as an example, the location coordinates of the distribution center and 10 customers, and the product demand of each customer are shown in Table 2.

At the same time, obtain the relevant receipt time window, unloading time, and stopover time in the international trade logistics center for statistics, as shown in Table 3.

Assuming the parameters corresponding to the traffic conditions in city A, the transport vehicles equipped in the distribution center are changed to Dongfeng Duolika transport vehicles (with a load capacity of 7 tons). Statistics are made on the number of transport vehicles required by these 10 distribution points. And taking into account the location coordinates of 10 customers, the demand for chilled meat, and the 7t load of refrigerated transport vehicles, the 10 customers are divided into the following 3 routes, as shown in Table 4.

Using Matlab 2011a calculation, decode the calculated solution space to get the optimal distribution route scheme. The results are shown in Table 5.

From the improved optimal route distribution table, we can see that after the improvement, the delay time in the logistics distribution process is basically 0, which can save time in the transportation process.

## 5. RFID Tags and Optimization Analysis

### 5.1. Modulation Mode Simulation

Different modulation methods can be achieved by changing the load impedance to change the current flowing through the antenna and the reflection coefficient of the antenna: ASK modulation can be achieved by changing the amplitude of the current, and PSK modulation can be achieved by changing the phase of the current. Under different modulation modes, the reflection coefficient of the tag is different, and the power entering the tag and the power reflected by the tag are different.  Figure 7 shows the Smith chart of reflection coefficients under different modulation modes.

Comparing the above four modulation methods, we can see the following:

1. Under ASK1 modulation, the available power entering the tag and the power reflected by the tag remain unchanged, which are 50% and 25%, respectively; under the other three modulation modes, the available power entering the tag decreases with the increase of the reflection coefficient.
2. PSK and ASK2 have the same tag useable power (83%) and reflected power (17%), but under ASK2 modulation, part of the tag useable power is consumed by extra resistors and cannot be used effectively.
3. ASK and PSK use nonlossy components to change the state of impedance, similar to PSK modulation. In the ideal case, the sum of the tag's available power and the tag's reflected power is a constant value. The tags of UHF RFID systems usually use load capacitance modulation to achieve ASK and PSK modulation from the tag to the reader. At this time, the power reflected by the tag is related to the modulation index and antenna loss, generally accounting for 10% to 20% of the total received power.

### 5.2. Tag Antenna Performance

By understanding the design of the tag antenna, we can see that the reduction or increase of the resonant frequency of the tag antenna can be achieved by adding capacitive or inductive loads. A capacitive load (low frequency) and an inductive load (high frequency) work together so that the tag antenna has two resonance modes, high and low. And the bandwidth of the S-parameter curve of the tag antenna can be changed by adjusting the length of the T-shaped microstrip structure and adjusting the depth of the U-shaped hollow structure. RFID tag antennas for metal backgrounds were designed and simulated using HFSS as shown in Figure 8.

It can be seen from the simulation results of the tag antenna that the two lowest points of the S-parameter curve of this tag antenna are 870 MHz and 915 MHz, respectively, and these two frequencies are also the resonant frequencies of the tag antenna.

The comparison between the measurement results of the tag antenna and the simulated junction impedance curve is shown in Figure 9. At 915 MHz, the antenna impedance obtained by simulation is (13.5∼120j) ohm, and the antenna impedance is (15.3∼123j) ohm obtained from the test, and the tag antenna and the tag chip are well matched.

### 5.3. Optimization Results

In order to have a general understanding of the optimization results of international trade logistics based on the Internet of Things technology proposed in this paper, this paper makes a rough simulation of the trade logistics of city A and analyzes it. It analyzes and compares the improvement effect of this paper with the effect before improvement and makes statistics on five different logistics distribution centers. It counts the amount of goods carried in the same time period to reflect the optimization effect of trade logistics. The specific situation is shown in Figure 10.

Through the above comparative analysis, we can see that after the improvement, the logistics has a relatively obvious increase in the carrying capacity. Before the improvement, the carrying capacity of site 1 was 15,000 tons, accounting for 12.93%; the carrying capacity of site 2 was 19,000 tons, accounting for 16.38%; the carrying capacity of site 3 was 26,000 tons, accounting for 22.41%; the carrying capacity of site 4 is 31,000 tons, accounting for 26.72%; and the carrying capacity of site 5 is 25,000 tons, accounting for 21.55%. On the other hand, for the improved carrying capacity, the carrying capacity of site 1 is 25,000 tons, accounting for 15.82%; the carrying capacity of site 2 is 29,000 tons, accounting for 18.35%; the carrying capacity of site 3 is 34,000 tons, accounting for 21.52%; the carrying capacity of site 4 is 38,000 tons, accounting for 24.05%; and the carrying capacity of site 5 is 32,000 tons, accounting for 20.25%.

Based on the above analysis, we can conclude that the improved international trade logistics has increased the carrying capacity by 34.2% and shortened the carrying time by 28.6%, which has been significantly improved.

## 6. Conclusions

This paper mainly studies the optimization design of international trade logistics based on the Internet of Things technology, through the optimization and improvement of RFID technology, and the key technology of the Internet of Things. Through its tracking and identification of a path in the process of trade logistics transportation, and optimizing it, the optimal transportation path can be achieved in the actual transportation process. This also fully guarantees the international trade carrying capacity, carrying capacity, and carrying efficiency. And in the experimental part, a simulation experiment is carried out on the optimization of its logistics, the results also show that the scheme is feasible. And in the analysis part, the relative RFID technology is compared and analyzed to explore the actual effect of its optimization.

## Figures and Tables

**Figure 1:** The structure of the Internet of Things.

**Figure 2:** Internet of Things technology system framework.

**Figure 3:** Basic composition of RFID.

**Figure 4:** Relationship between received signal power and distance under the two models.

**Figure 5:** Label equivalent circuit.

**Figure 6:** International logistics barriers.

**Figure 7:** Reflection coefficients of labels under four different modulation modes.

**Figure 8:** The frequency correspondence between the T-shape and U-shape of the S-parameter curve of the tag antenna.

**Figure 9:** Comparison of measurement results of tag antenna resistance and reactance with simulation results.

**Figure 10:** Comparison of logistics carrying capacity before and after optimization.

**Table 1:** Collected data and equipment used.

Numbering	Link	Collected data	Equipment
1	Discharge	Distribution vehicle situation, cargo situation, distribution center information	RFID reader, measuring instrument information
2	Sales and processing	Workshop information, operating hours, operators, packaging information	RFID reader, video capture
3	Sales	Product information	RFID reader, barcode

**Table 2:** Statistical table of customer coordinates and product demand.

Serial number	*X* coordinate	*Y* coordinate	Demand
0	13426.14	2893.12	0
1	13462.11	2894.16	1
2	13428.16	2897.36	1.2
3	13422.62	2894.19	2
4	13429.18	2894.43	2
5	13481.64	2896.36	3.5
6	13492.11	2891.18	2
7	13466.23	2899.48	1
8	13428.36	2894.18	0.5
9	13492.16	2895.77	2.5
10	13411.12	2894.61	1.5

**Table 3:** Receipt time window, unloading time, and dwell time statistics.

Serial number	Earliest pickup time	Latest pickup time	Dwell time
0	6:00	17:30	0
1	7:15	14:30	0.5
2	6:00	15:30	0.75
3	7:00	16:00	0.25
4	7:00	10:30	0.25
5	6:30	8:00	0.75
6	6:45	13:00	0.5
7	6:45	10:30	0.5
8	6:30	17:15	0.33
9	6:00	12:00	0.5
10	6:00	15:00	0.25

**Table 4:** Route division table.

Vehicle serial number	Customer point	Number of customers	Vehicle capacity
1	1, 2, 4, 7, 8	5	6
2	5, 9	2	6
3	3, 6, 10	3	5.5

**Table 5:** Optimal route delivery table.

Vehicle serial number	Shipping order	Number of customers	Delivery mileage	Waiting time	Delay time
1	0-7-2-8-4-1-0	5	13.47	0	0
2	0-5-9-0	2	21.09	0	0
3	0-9-30-26-23-0	3	17.82	0	0

## Data Availability

No data were used to support this study.
